# Luteolin Induced Hippocampal Neuronal Pyroptosis Inhibition by Regulation of miR-124-3p/TNF-*α*/TRAF6 Axis in Mice Affected by Breast-Cancer-Related Depression

**DOI:** 10.1155/2022/2715325

**Published:** 2022-05-06

**Authors:** Qing Zhu, Pan Meng, Yuanshan Han, Hui Yang, Qin Yang, Zhuo Liu, Yuhong Wang, Minghui Long

**Affiliations:** ^1^Science and Technology Innovation Center, Hunan University of Chinese Medicine, Changsha, Hunan Province 410208, China; ^2^Hunan Cancer Hospital/The Affiliated Cancer Hospital of Xiangya School of Medicine, Central South University, Changsha, Hunan 410013, China; ^3^The First Affiliated Hospital, Hunan University of Chinese Medicine, Changsha, Hunan 410007, China

## Abstract

**Background:**

Breast-cancer-related depression (BCRD) is associated with an increased mortality rate among breast cancer (BC) survivors. Luteolin has many pharmacological effects, particularly in the treatment of BC. In this study, we aimed to explore the anti-BCRD activity of luteolin and its underlying functional mechanism.

**Methods:**

A BCRD mouse model was induced by injecting 4T1 cells and corticosterone (COR). Behavioral test, terminal deoxynucleotidyl transferase dUTP nick end labeling (TUNEL) staining, Nissl staining, immunofluorescence, reverse-transcription quantitative PCR (RT-qPCR), and western blotting were used to study the effect of luteolin in mice with BCRD in vivo. A COR-induced neuron injury model was established in HT-22 cells in vitro. The role of miR-124-3p in the anti-BCRD effects of luteolin was studied using a miR-124-3p inhibitor.

**Results:**

Luteolin significantly reduced the size and weight of the tumor, increased the mice entry frequency in the symmetrical sector, and reduced the duration of immobility in the tail suspension and forced swimming tests of mice affected by BCRD. Simultaneously, apoptosis of hippocampal neurons was inhibited, and the number of Nissl bodies increased with luteolin treatment. In addition, luteolin resulted in the upregulation of miR-124-3p expression in the hippocampus and downregulated the expression of tumor necrosis factor-*α* (TNF-*α*) and TNF receptor-associated factor 6 (TRAF6), as well as lowered the phosphorylation levels of nuclear factor-kappa B (NF-*κ*B) and IkappaB (I*κ*B). Luteolin also inhibited pyroptosis of hippocampal neurons in mice affected by BCRD, as revealed by the low protein levels of NOD-like receptor protein 3 (NLRP3), caspase-1, gasdermin D-N (GSDMD-N), interleukin (IL)-1*β*, and IL-18. However, the miR-124-3p inhibitor significantly reversed the therapeutic effect of luteolin on COR-induced HT-22 cells.

**Conclusion:**

Our study demonstrated that the anti-BCRD function of luteolin was mediated by regulating the miR-124-3p/TNF-*α*/TRAF6-related pathway and inhibiting neuronal cell pyroptosis and subsequent inflammation. Therefore, luteolin may be a potential drug candidate in the treatments of BCRD.

## 1. Background

Breast cancer (BC) is the most common malignant tumor and the main cause of cancer-related deaths among patients worldwide [1]. Depression is an emotional disorder common among patients with cancer. BC patients have the highest incidence and most severe depression [2]. Previous studies have shown that depression is associated with increased mortality in BC patients [3]. Therefore, the prevention and treatment of depression are key to improving the life quality and expectancy of BC patients [4].

Neuroinflammation and oxidative stress are important factors leading to depression and cognitive impairment in patients with BC [5]. Kim et al. found through blood analysis that depression in BC patients was closely correlated with the imbalance of proinflammatory factors and anti-inflammatory factors, such as tumor necrosis factor-*α* (TNF-*α*) [6]. At present, most researches on the mechanism of breast cancer-related depression (BCRD) focus on apoptosis or necrosis of hippocampal neurons caused by inflammation. The growth and treatment of tumors can cause significant changes in hippocampal volume and decreased neurogenesis, thereby resulting in depression [7]. Research has shown the development of depression to be related to pyroptosis mediated by NOD-like receptor protein 3 (NLRP3) [8]. Pyroptosis is a caspase-1-dependent programmed cell death pathway that is closely related to inflammation and is widely associated with central nervous system diseases [9]. It was found that TNF-*α*, a proinflammatory cytokine, could activate caspase-1 in upper 3T3-L1 cells [10]. At the same time, it can activate caspase-1 and other factors by mediating multiple inflammatory signaling pathways and lead to neuronal pyroptosis [8, 11].

MicroRNAs (miRNAs) are small noncoding RNA molecules that play a significant role in regulating the expression of genes related to the inflammatory response [12]. For instance, miRNA-495-3p inhibits inflammation and apoptosis in human nucleus pulposus cells by targeting the IL5RA pathway [13]. MiR-21 directly targets A20, promotes the activation of NLRP3 inflammatory corpuscles, and influences pyroptosis in lipopolysaccharide (LPS) induced sepsis in mice [14]. MiR-124-3p is one of many miRNAs that can inhibit neuronal inflammation [15]. Research has also shown that miR-124-3p is associated with a poor prognosis of BC [16]. In addition, miR-124-3p targets the TNF receptor-associated factor 6 (TRAF6) mRNA, which reduces the production of inflammatory cytokines induced by LPS and inhibits p38 mitogen-activated protein kinase (MAPK) and nuclear factor-kappa B (NF-*κ*B) signaling pathway activation, as well as weakens severe community-acquired pneumonia [17].

Luteolin is a natural flavonoid compound with protective effects against many diseases. It inhibits tumor proliferation by upregulating miR-124-3p, thus inducing MAPK activation [18]. Luteolin can also significantly reduce the growth and epithelial-mesenchymal transition (EMT) of BC cells and exert antitumor effects [19]. In addition, luteolin can play anti-inflammatory and neuroprotective roles in microglia by regulating its activation [20]. Luteolin also induces upregulation of miR-132, thereby promoting neuronal survival and neurite growth and exerting neurotrophic effects [21]. These findings lead us to speculate that luteolin might affect the pyroptosis pathway of hippocampal neurons by regulating the miR-124-3p/TNF-*α*/TRAF6 axis, thus relieving BCRD.

To verify this hypothesis, we used 4T1 cells and corticosterone (COR) to induce simulated BCRD in mice. We observed the effects of luteolin on tumor development, depressive behavior, and the cascade reaction of miR-124-3p/TNF-*α*/TRAF6 in the hippocampus and modulation of pyroptosis by NLRP3. Luciferase assays detected the targeted binding between miR-124-3p and TRAF6. Finally, an miR-124-3p inhibitor was used to further evaluate the role of miR-124-3p in luteolin-related anti-BCRD effects.

## 2. Methods

### 2.1. Construction of BCRD Animal Model

Female BALB/c mice were purchased from Hunan Slack Jingda Experimental Animal Co. Ltd. (experimental animal license number: SCXK (Xiang) 2013-0004, certificate number: 43004700028075). Before the experiments were conducted, the mice were housed in an animal room and provided food and water for 10 days.

The 4T1 inflammatory BC cell line was obtained from Abiowell Co. Ltd., and its growth state was observed under a microscope (DSZ2000X; Beijing Zhongxian Hengye Instrument co. Ltd., China). The cells were cultured in Dulbecco's modified eagle medium (DMEM) supplemented with 10% fetal bovine serum and 1% penicillin-streptomycin. The cultures were maintained in a humidified atmosphere containing 5% CO_2_ at 37°C and then harvested using trypsin‐EDTA (Invitrogen, USA). Finally, 1 × 10^7^ cells were diluted in phosphate-buffered saline (PBS) and injected subcutaneously into the right mammary fat pads of female BALB/c mice. After 7 days, tumor formation was observed, and the BC model was successfully established. Then, the COR suspension (30 mg/kg) was injected subcutaneously into BC mice for 21 days. A compound animal model of BC combined with depression was established.

### 2.2. Animal Treatments

The experimental groups included the control, BCRD, positive drug (paclitaxel + fluoxetine), and luteolin groups, with five mice in each group. In addition to the control group, the other groups of mice received BCRD model replicas. Moreover, luteolin group mice received intraperitoneal injection of luteolin at a dose of 50 mg/kg/d [22]. The positive drug group mice were injected with paclitaxel liposomes intraperitoneally at a dose of 20 mg/kg once a week and fluoxetine hydrochloride by gastric gavage at a dose of 7.8 mg/kg/d. These drugs were administered for 21 consecutive days.

### 2.3. Open-Field Experiment

Before the test, all the mice were fasted for 24 h and placed in the center of an open field consisting of a square wooden arena (40 × 60 × 50 cm), with the inner walls covered with black surfaces. The number of times each mouse entered the symmetric sector within 6 min was counted by trained observers who were blinded to the experimental group [23].

### 2.4. Tail Suspension Test (TST)

Before the test, all mice were fasted for 24 h and suspended (hung upside down) by their tails (1–2 cm from the tail tip) at 60 cm above the ground. Each mouse was separated from the others by a certain distance. After 30 s of adaptation, the limb immobility duration of each mouse was recorded for 3 min.

### 2.5. Forced Swimming Test (FST)

In this experiment, the mice were forced to swim in a water tank with no escape [24]. Each mouse was placed for 6 min in a glass cylinder (30 cm height and 10 cm diameter) filled with water up to a height of 25 cm at 25 ± 1°C to record the immobility duration. The mice were considered to be immobile when they stopped swimming and did nothing except the necessary actions to keep their head above the water.

### 2.6. Cell Culture and Transfection

Hippocampal neuron cell line (HT-22), obtained from Abiowell Co. Ltd., was maintained in DMEM and incubated in a 5% CO_2_ incubator at 37°C. These cells were divided into three groups: control, COR, and COR + luteolin. The COR and COR + luteolin groups were treated with 200 *μ*M COR for 24 hours. In addition, cells in the COR + luteolin group were treated with 20 *μ*M luteolin for 24 h [20].

The Lipofectamine 2000 transfection reagent (11668019, Invitrogen) was used for transient transfection of miR-124-3p inhibitor and the corresponding negative control (NC) into the HT-22 cells. The cells were grouped as follows: control, COR, COR + luteolin, COR + luteolin + NC inhibitor, and COR + luteolin + miR-124-3p inhibitor.

### 2.7. Reverse-Transcription Quantitative PCR

The total RNA from cells or mice hippocampal tissue was extracted using TRIzol reagent (Invitrogen) and reversely transcribed to cDNA using the mRNA reverse transcription kit (CW2569, CWBIO, China) according to the manufacturer's instructions. Reverse-transcription quantitative PCR (RT-qPCR) detection was conducted at 95°C for 10 min, 95°C for 15 s, and 60°C for 30 s, 40 cycles. The 2^−ΔΔct^ method was used to analyze the expression of TRAF6 and miR-124-3p, as described in a previous study [25]. *β*-Actin and U6 were used as endogenous controls. The primer sequences are shown in Table 1.

### 2.8. Western Blotting

Proteins were resolved from the cells and mice hippocampal tissue using RIPA buffer (AWB0136a, Abiowell, China) by following the manufacturer's instructions. The proteins were divided using 10% (w/v) acrylamide gel SDS-PAGE and transferred to a nitrocellulose membrane. After blocking with 5% bovine serum albumin for 2 h at room temperature, immunoblotting was performed using TNF-*α* (ab6671; Abcam, UK), phosphorylated NF-*κ*B (p-NF-*κ*B; ab76302; Abcam), NF-*κ*B (ab32536; Abcam), IkappaB (I*κ*B; ab32518; Abcam), phosphorylated I*κ*B (p-I*κ*B; ab133462; Abcam), NLRP3 (ab263899; Abcam), caspase-1 (22915-1-AP; Proteintech, USA), GSDMD-N (ab215203; Abcam), IL-1*β* (16806-1-AP; Proteintech), IL-18 (ab191860; Abcam), or *β*-actin (60008-1-Ig; Proteintech). *β*-Actin was used as an internal control. The membrane was then incubated with the HRP-bound secondary antibody. Finally, the proteins were incubated with SuperECL Plus (Advansta, USA) for 5 min. They were visualized using the chemiluminescence imaging system (ChemiScope 6100, Guangzhou Qinxiang, China). The gray value was analyzed and calculated using ImageJ software.

### 2.9. Luciferase Reporter Assays

293A cells were purchased from HonorGene and cotransfected using Lipofectamine 2000 with pHG-MirTarget-TRAF6-3U plasmid and miRNA negative control or mmu-miR-124-3p mimics and pHG-MirTarget-TRAF6 MUT-3U plasmid and miRNA negative control or mmu-miR-124-3p mimics. After 24 h, following cell collection, luciferase activity was evaluated using dual-luciferase reporter assay system (E1910, Promega, USA).

### 2.10. Terminal Deoxynucleotidyl Transferase dUTP Nick End Labeling (TUNEL) Staining

The collected hippocampal tissue was fixed in 4% paraformaldehyde, dehydrated, embedded in paraffin, and sectioned. Then, the slices were baked at 60°C for 12 h and dewaxed. Following the TUNEL Kit (KGA7053, KeyGEN Biotech Co. Ltd., China) illustrations, the samples were incubated with 50 *μ*L endogenous avidin-blocking solution A and 50 *μ*L endogenous avidin-blocking solution B for 20 min, respectively. Subsequently, the buffer with TDT enzyme was used to incubate the samples in the dark for 60 min at 37°C. The nucleus was stained with DAPI. Finally, a fluorescence microscope (BA410E, Motic, China) was used to observe and collect images.

### 2.11. Nissl Staining

The tissue slices were dewaxed and hydrated as described previously [26]. The sections were then placed in Nissl staining solution (Wellbio, China) for 1 min., sealed with glycerin, and observed under a microscope (Motic, China).

### 2.12. Immunofluorescence (IF)

The tissues were fixed in 4% paraformaldehyde, embedded in paraffin, and sectioned. HT-22 cells were fixed on glass slides with 4% paraformaldehyde. The tissue slices and cells slides were incubated with the primary antibody NeuN (ab177487; Abcam) and caspase-1 (MA5-16215; Thermo Fisher) overnight at 4°C. The secondary antibody of anti-rabbit (SA00013-2; Proteintech) and anti-mouse-IgG (SA00013-3; Proteintech) was applied the next day. DAPI solution (AWC0291a; Abiowell, China) was used to stain the nucleus of the cells. A fluorescence microscope was used to assess the stained results.

### 2.13. Cell Counting Kit-8 (CCK8) Assay

The cells in the logarithmic growth stage were digested and counted. They were then seeded into 96-well plates at a density of 5 × 10^3^ cells/well, 100 *μ*L per well. After 24 h, the cells were treated according to the groups mentioned above (control, COR, and COR + luteolin). CCK8 solution of 10 *μ*L (AWC0114a; Abiowell, China) was added to each well. A BioTek enzyme plate analyzer (MB-530; HEALES, China) was used to determine the absorbance at 450 nm.

### 2.14. Immunocytochemistry

The slides of cells were fixed with 4% paraformaldehyde and then repaired using 10 mM sodium citrate (pH 6.0). After removing endogenous peroxidase with 3% H_2_O_2_, the sample was incubated overnight with primary antibody GSDMD-N (20770-1-AP; Proteintech) at 4°C. Next, the sample was incubated with secondary antibody anti-rabbit-IgG antibody-HRP polymer at 37°C for 30 min. DAB solution was dripped and stained with hematoxylin. The slices were placed in xylene, dehydrated using a concentration gradient of ethanol, and sealed with neutral gum. A microscope was used to observe and collect the images.

### 2.15. Statistical Analysis

GraphPad Prism 8 software (GraphPad Inc., USA) was used for statistical analysis of the data. The statistical significance was determined by a nonpaired *t*-test between the two groups. One-way analysis of variance (ANOVA) was used to define three or more groups. The data were expressed as mean ± standard deviation (SD). *P* < 0.05 indicated a significant difference between the results.

## 3. Results

### 3.1. Luteolin Alleviated the BCRD Symptoms in the Affected Mice

To study the effect of luteolin on BCRD, we established a mouse model of BCRD. Tumor formation occurred in all groups, except the control group (Figure 1(a)). Compared to the BCRD group, in the paclitaxel + fluoxetine and luteolin groups, the tumor volume and weight decreased (Figures 1(b)–1(c)). These results indicated that the positive drugs (paclitaxel + fluoxetine) and luteolin had certain therapeutic effects on mice affected by BCRD. Subsequently, we conducted behavioral tests on these mice. The number of times the BCRD group mice entered the symmetric sector was markedly lower than that of the control group (Figure 1(d)). In contrast, these symptoms were relieved after treatment with paclitaxel + fluoxetine or luteolin. Similarly, the TST and FST experiments observed that the static time of mice in the BCRD group increased, whereas that of mice treated with paclitaxel + fluoxetine or luteolin decreased (Figures 1(e)–1(f). The above results suggested that BCRD group mice had depressive behavior and evidently be improved by luteolin.

### 3.2. The Protective Effect of Luteolin on Hippocampal Neurons

The development of BCRD is closely associated with nerve injury. TUNEL staining showed that compared to the control group, the BCRD group had a significantly higher number of TUNEL-positive cells. However, after treatment with paclitaxel + fluoxetine or luteolin, the apoptosis was significantly reversed (Figure 2(a)). Nissl staining analysis validated that hippocampus neurons of the control group were closely arranged, their cell structure was visible, and Nissl corpuscles were abundant. In contrast, the hippocampal neurons of the BCRD group were loosely arranged; the outline of their cells was blurred and atrophied; and the number of Nissl corpuscles was markedly lower (Figure 2(b)). The above results showed that hippocampal neurons in mice affected by BCRD were severely injured. However, after treatment with paclitaxel + fluoxetine or luteolin, the state of hippocampal neurons was alleviated.

### 3.3. Luteolin Inhibited Pyroptosis of Hippocampal Neurons

We tested the effects of luteolin on hippocampal neuronal pyroptosis. The coexpression of caspase-1 and NeuN was evaluated by IF. The results showed that the expression of active caspase-1 positive neurons in the hippocampus was significantly increased in BCRD group mice compared to that in the control group. However, it was significantly decreased after treatment with paclitaxel + fluoxetine or luteolin (Figure 3(a)). In addition, western blotting results were consistent with those of IF (Figure 3(b)). They showed that the levels of NLRP3, caspase-1, GSDMD-N, IL-1*β*, and IL-18 in the hippocampus of BCRD group mice were significantly high. However, after treatment with paclitaxel + fluoxetine or luteolin, the levels of these proteins decreased significantly (Figure 3(b)). These results suggest that luteolin may possibly alleviate hippocampal neuron injury in mice affected by BCRD by inhibiting pyroptosis and subsequent inflammation.

### 3.4. Luteolin Effects on miR-124-3p/TNF-*α*/TRAF6 Axis in Hippocampal Neurons

To examine luteolin's mechanism in the regulation of BCRD in mice, we tested the expression of miR-124-3p/TNF-*α*/TRAF6 axis-related factors. RT-qPCR results detected that miR-124-3p was diminished considerably, and TRAF6 was augmented markedly in the hippocampus of BCRD group mice. These expressions were reversed after paclitaxel + fluoxetine or luteolin treatment (Figure 4(a)). Meanwhile, western blotting results showed that TNF-*α* levels in the hippocampus decreased significantly in BCRD group mice compared to those in the control group. In contrast, TNF-*α* levels increased substantially after treatment with paclitaxel + fluoxetine or luteolin (Figure 4(b)). In addition, we detected that the expression of p-NF-*κ*B and p-I*κ*B was augmented in the BCRD group, but these expressions reversed after treatment with paclitaxel + fluoxetine or luteolin (Figure 4(b)). Using bioinformatics analysis, we found that miR-124-3p and TRAF6 targeted binding sites. A double luciferase assay verified the targeting relationship between miR-124-3p and TRAF6 (Figure 4(c)). These results suggest that luteolin may affect pyroptosis and inflammation of hippocampal neurons in mice affected by BCRD via the miR-124-3p/TNF-*α*/TRAF6 axis.

### 3.5. Luteolin Inhibited the Pyroptosis of HT-22 Cells Stimulated by Corticosterone

We used COR to induce the neuron injury model of HT-22 cells in vitro. Compared with the control group, the cell viability was decreased significantly by COR treatment but increased after luteolin treatment (Figure 5(a)). Immunocytochemistry examination showed that the expression of caspase-1 in the COR group was considerably upregulated compared to that in the control group, but the expression was significantly reversed after luteolin treatment (Figure 5(b)). GSDMD-N levels were investigated by IF (Figure 5(c)). The results showed that GSDMD-N levels in the COR group were substantially higher than those of the control group, but the expression was reversed after luteolin treatment. These results suggest that after COR treatment, HT-22 cells were induced to pyroptosis, but these conditions were improved after luteolin treatment.

### 3.6. Luteolin Inhibited HT-22 Cell Pyroptosis through miR-124-3p/TNF-*α*/TRAF6 Axis

To further elucidate the miR-124-3p/TNF-*α* axis in protecting neurons from pyroptosis, NC and miR-124-3p inhibitors were transfected into HT-22 cells. RT-qPCR results detected that miR-124-3p had a good inhibitory efficiency. Moreover, when miR-124-3p was inhibited, TRAF6 mRNA expression was upregulated significantly (Figure 6(a)). Western blotting results observed that the miR-124-3p inhibitor reversed the COR-induced upregulation of TNF-*α* expression and the inhibition of p-NF-*κ*B and p-I*κ*B expression in HT-22 cells mediated by luteolin (Figure 6(b)). Subsequently, we determined the levels of pyroptosis-related proteins. The results indicated that the miR-124-3p inhibitor significantly improved the inhibitory effect of luteolin on the COR-induced increase in the levels of pyroptosis-related proteins (NLRP3, caspase-1, GSDMD-N, IL-1*β*, and IL-18) in HT-22 cells (Figure 6(c)). To summarize, luteolin inhibited the HT-22 cell pyroptosis through miR-124-3p/TNF-*α*/TRAF6 axis.

## 4. Discussion

Depression is an important complication of BC and is associated with high mortality [27, 28]. BCRD has become a research hotspot in recent years. In this study, we established a simulated BCRD mouse model by injecting 4T1 cells and COR. Tumors appeared in the BCRD group mice. In the open field experiment, the number of times the BCRD group mice entered the symmetrical sectors reduced, indicating that they had lost interest in exploring new environments. The increase in immobility duration during the TST and FST has been interpreted as an indicator of depression [29]. Our results showed that the immobility duration of BCRD group mice increased significantly during the TST and FST. These results indicated that the BCRD model was successfully established.

Increasing evidence has shown that the flavonoid luteolin has anti-inflammatory, anticancer, antianxiety, and memory improvement effects [30, 31]. For example, a study showed that luteolin can induce apoptosis in BC cells [32]. Another study revealed that luteolin exerts antidepressant effects by inhibiting endoplasmic reticulum stress [22]. Our study found that after luteolin treatment, tumor volume and weight in BCRD group mice were reduced significantly and depressive behavior was alleviated considerably. These effects were consistent with those observed in the positive drug (paclitaxel + fluoxetine) group. In addition, we detected neuronal damage in the BCRD group mice and found that luteolin treatment significantly reversed the decrease of Nissl bodies and increase in neuronal apoptosis. This is consistent with previous studies [33]. These observations suggest that luteolin might have certain relieving effects on BCRD.

Pyroptosis is a form of neuronal cell death [34]. Unlike other neuronal death mechanisms, pyroptosis is mediated by caspase-1, activated by inflammatory corpuscle NLRP3, and sheared GSDMD to form its N-terminal fragment. With the formation of pathological pores and cell rupture, pyroptosis induces the release of proinflammatory cytokines (IL-1*β* and IL-18), which further aggravates the inflammatory injuries [35, 36]. In this study, we found that the levels of pyroptosis-related proteins (NLRP3, caspase-1, and GSDMD-N) in hippocampal neurons and levels of inflammatory factors (IL-1*β* and IL-18) in the BCRD group mice increased significantly. After luteolin treatment, the levels of these related proteins decreased significantly, which was consistent with those of the positive control group. In vitro studies also showed that luteolin reduced the protein expression of caspase-1 and GSDMD-N in COR-stimulated neurons. Therefore, our results suggested that luteolin may alleviate BCRD symptoms by inhibiting neuronal pyroptosis.

MiR-124-3p is a member of the miRNA family responsible for regulating gene expression in various biological processes, including immunity and inflammation [37]. MiR-124-3p directly targets TRAF6 and inhibits the activation of the NF-*κ*B pathway [38]. In this study, TRAF6 expression was upregulated after inhibition of miR-124-3p. Meanwhile, the luciferase experiment revealed that miR-124-3p combined with TRAF6 in a targeted manner, which confirmed that miR-124-3p had a regulatory effect on TRAF6. It has been proposed that the miR-124-3p/TRAF6/TNF-*α* axis regulates pyroptosis. For instance, miR-124-3p can inhibit the activation of the inflammatory corpuscle NLRP3 by targeting TRAF6 [39]. TRAF6 promotes the oligomerization of NLRP3 and interaction between NLRP3 and apoptosis-related spot proteins including CARD [40]. Our work found that the expression of miR-124-3p was downregulated and that of TRAF6 and TNF-*α* was upregulated, and the NF-*κ*B pathway was activated in BCRD group mice. These results supported the key role of the miR-124-3p/TRAF6/TNF-*α* axis in BCRD. In addition, luteolin reversed the expression of miR-124-3p, TRAF6, and TNF-*α* in BCRD group mice and inhibited NF-*κ*B pathway activation. However, in vitro studies showed that miR-124-3p inhibition could reverse the therapeutic effect induced by luteolin, reflecting the requirement of luteolin-related antidepression activity on the activation of miR-124-3p. These data further highlighted the key role of miR-124-3p in BCRD treatment.

## 5. Conclusions

Our research concludes that luteolin can effectively reduce tumor development and depression-like behavior in mice affected by BCRD. This effect of luteolin can be related to its protective effect on pyroptosis in hippocampal neurons. The mechanism of action includes the regulation of the miR-124-3p/TRAF6/TNF-*α* axis by luteolin. These results supported the interest in luteolin-based treatment strategies and further development of complementary drugs to treat BCRD.

## Figures and Tables

**Figure 1:** Luteolin alleviated the BCRD symptoms in the affected mice: (a) representative images of the tumor, (b) tumor volume, (c) tumor weight, (d) open-field experiment, (e) tail suspension test, and (f) forced swimming test. ^∗^ – compared to the control group. ^#^ – compared to the BCRD group. *p* < 0.05.

**Figure 2:** The protective effect of luteolin on hippocampal neurons: (a) TUNEL staining and (b) Nissl staining. ^∗^ – compared to the control group. ^#^ – compared to the BCRD group. *p* < 0.05.

**Figure 3:** Luteolin inhibited pyroptosis of hippocampal neurons: (a) the protein expression of caspase-1 and NeuN detected using immunohistochemistry (400×) and (b) the protein levels of NLRP3, caspase-1, GSDMD-N, IL-1*β*, and IL-18 detected using western blotting. ^∗^ – compared to the control group. ^#^ – compared to the BCRD group. *p* < 0.05.

**Figure 4:** Luteolin effects on miR-124-3p/TNF-*α*/TRAF6 axis in hippocampal neurons: (a) RT-qPCR detected relative expression of miR-124-3p and TRAF6 and (b) the expression of TNF-*α*, NF-*κ*B, p-NF-*κ*B, I*κ*B, and p-I*κ*B detected by western blotting. ^∗^ – compared to the control group. ^#^ – compared to the BCRD group. *p* < 0.05. (c) Website predicted target sequence of miR-124-3p and TRAF6. The targeting relationship between miR-124-3p and TRAF6 verified by luciferase assay. ^∗^ – compared to the NC group. *p* < 0.05.

**Figure 5:** Luteolin inhibited the pyroptosis of HT-22 cells stimulated by corticosterone: (a) the cell viability was observed by CCK8 and (b) immunocytochemistry examination to show the expression of caspase-1, (c) IF evaluated the GSDMD-N level. ^∗^ – compared to the control group. ^#^ – compared to the COR group. *p* < 0.05.

**Figure 6:** Luteolin inhibited HT-22 cell pyroptosis through miR-124-3p/TNF-*α*/TRAF6 axis: (a) miR-124-3p and TRAF6 levels detected by RT-qPCR; (b) the expression of TNF-*α*, NF-*κ*B, p-NF-*κ*B, I*κ*B, and p-I*κ*B evaluated by western blotting; and (c) the protein expression of NLRP3, caspase-1, GSDMD-N, IL-1*β*, and IL-18 detected by western blotting. ^∗^ – compared to the control group. ^#^ – compared to COR group. & – compared to the COR + luteolin + NC inhibitor group. *p* < 0.05.

**Table 1:** Primer sequences.

Gene	Sequences (5′-3′)
TRAF6	F: ATTGACAGCCACCTCCCCT
	R: TTGGCGTCCATGACCTCTTC

miR-124-3p	F: TGCGTGT TCACAGCGGA CCTT
	R: GCTGTCAACGATACGCTACGTAA

*β*-actin	F: ACATCCGTAAAGACCTCTATGCC
	R: TACTCCTGCTTGCTGATCCAC

U6	F: CTCGCTTCGGCAGCACA
	R: AACGCTTCACGAATTTGCGT

## Data Availability

The data used to support the findings of this study are available from the corresponding author upon request.
